The article "microRNA-195 attenuates neuronal apoptosis in rats with ischemic stroke through inhibiting KLF5-mediated activation of the JNK signaling pathway" was retracted in 2023. Reasons: results that could not be reproduced; concerns about the data.

# microRNA-195 attenuates neuronal apoptosis in rats with ischemic stroke through inhibiting KLF5-mediated activation of the JNK signaling pathway

**DOI:** 10.1186/s10020-020-00150-w

**Published:** 2020-04-09

**Authors:** Lisha Chang, Wan Zhang, Songxin Shi, Yanbo Peng, Dali Wang, Li Zhang, Jiang Zhang

**Affiliations:** 1 Department of Neurology, North China University of Science and Technology Affiliated Hospital, No. 73, Jianshe South Road, Tangshan, 063000 Hebei Province People’s Republic of China; 2 Quality Control Office, North China University of Science and Technology Affiliated Hospital, Tangshan, 063000 People’s Republic of China

**Keywords:** microRNA-195, KLF5, JNK signaling pathway, Ischemic stroke, Apoptosis, Plasticity

## Abstract

**Background:**

Accumulating evidence has implicated the regulation of microRNAs (miRs) in ischemia stroke. The current study aimed to elucidate the role of microRNA-195 (miR-195) in neuronal apoptosis and brain plasticity in rats with ischemic stroke via the JNK signaling pathway/KLF5 axis.

**Methods:**

Ischemic stroke rat models were established by middle cerebral artery occlusion (MCAO), and oxygen deprivation (OGD) models were constructed in rat neuronal cells, followed by gain- or loss-of-function of miR-195 and/or KLF5 in rats and cells. Infarct volume, neuronal loss and ultrastructure, the expression of GAP-43, SYP and KLF5 protein as well as cell apoptosis were determined in the rats. Caspase-3 activity as well as the expression of miR-195, KLF5, GAP-43, SYP, JNK, phosphorylated JNK, Bax and Bcl-2 was measured in the cells.

**Results:**

The infarct size, expression of GAP-43 and SYP protein and apoptotic cells were increased in the miR-195^−/−^ MCAO rats, while reductions were detected in the miR-195 mimic MCAO and KLF5^−/−^ MCAO rats. Bcl-2 expression was increased, Bax and Caspase-3 expression as well as the ratio of phosphorylated JNK/JNK was decreased in response to miR-195 overexpression or KLF5 knockdown. Interestingly, the silencing of KLF5 reversed the effects exerted by the miR-195 inhibitor on the expression of Bcl-2, phosphorylated JNK/JNK, Bax and Caspase-3.

**Conclusions:**

Collectively, our study unraveled that miR-195 could down-regulate KLF5 and block the JNK signaling pathway, ultimately inhibiting neuronal apoptosis in rats with ischemic stroke.

## Background

Stroke remains a chief contributor to physical disability, and also one of the fatal causes of death globally, with about 17 million diagnosed cases annually (Sun et al. 2016). Stoke is cerebrovascular interruption of blood supply to region of the brain that is originated from ischemia or hemorrhage, with ischemia stroke representing approximately 87 % of all stroke cases (Rink and Khanna 2011). In the event of insufficient blood-supply to a region of the brain, ischemia stroke can trigger a series of pathological events in a few minutes after the onset of the disease, ultimately resulting in irreversible neuronal injury (Sorensen et al. 2014). Ischemic stroke consists of a number of heterogeneous disorders as a result from genetic and environmental risk factors (Liu et al. 2014). Thrombolytic therapy and rehabilitation exercise therapy have proved to be effective treatment methods for ischemic stroke, helping to accelerate cerebral blood flow and patient recovery (Tian et al. 2013). However, the cellular and molecular mechanisms by which stroke promotes cell apoptosis and neurological dysfunction remain unclear.

Non-coding RNAs, such as microRNAs (miRs), are significant regulatory factors for both tissue developments and diseases owing to their function as translational repressors (Selvamani et al. 2012). Numerous miRs have been found to be closely related to ischemic stroke, including that of miR-124 and miR-134 (Sun et al. 2013, Spinato et al. 2014). Huang et al. concluded that miR-195 acts as a vasculogenesis suppresser in brain arteriovenous malformations (Huang et al. 2017). Moreover, it has been found that in chronic brain hypoperfusion, miR-195 could potentially regulate dendritic degeneration and neuronal death (Chen et al. 2017). Sp1-like transcription factors, Kruppel-like factors (KLFs), are involved in many cellular processes, such as embryonic development, cell proliferation and differentiation (Nandan et al. 2010). As a factor of the KLFs family, KLF5 could characteristically promote the proliferation of normal cells and tumor cells such as breast cancer, and intestinal tumorigenesis (Nandan et al. 2010, Tetreault et al. 2013). Besides, KLF5 not only was expressed at a high level in the walls of unruptured giant human cerebral aneurysms but also accelerated macrophage infiltration (Nakajima et al. 2012). Existing literature has suggested that miRs are capable of modulating angiotensin II-stimulated endothelial inflammation and migration (Zhu et al. 2011). Moreover, angiotensin II can elevate the extent of KLF5 phosphorylation and promote its communication with c-Jun (Paragas et al. 2009). c-Jun N-terminal kinases (JNKs) have shown their prominent roles in numerous diseases including laryngeal cancer, human colon cancer, neuro-degeneration (Wang et al. 2015) (Bogoyevitch et al. 2010, Gao et al. 2016). A previous study revealed that suppression of JNK protects neuronal cell against excitotoxic damage in rat models of cerebral ischemia (Coffey 2014). The current study aimed to obtain evidence illustrating the molecular mechanism by which miR-195 influences ischemic stroke as well as its underlying molecular mechanism.

## Methods

### Model induction

Wild-type Sprague Dawley (SD) male rats, miR-195 knockout (miR-195^−/−^) SD male rats and KLF5 knockout (KLF5^−/−^) male rats (12 rats in each) were all purchased from the Jackson Laboratory (Bar Harbor, ME, USA). The rats were allowed to acclimatize for one week in the animal facility before any intervention. The rats were granted with free access to water and food and housed under conditions with humidity of 60–70% with a 12/12 h day/night cycle at 22–24 °C. Middle cerebral artery occlusion (MCAO) rat models were induced by the suture method as previously reported by Zea Longa. Next, 1% pentobarbital sodium (4 mL/kg) was injected into the abdominal cavity of the rats for anesthesia. The rats were fixed in a supine position on the operating table. After hair removal by shaving, the rats were incised along the midline of carotid artery (CA). The right CA (CCA) and the external CA (ECA) were exposed and separated from the deep part of the muscles avoiding the injury of the vagus nerve and the internal carotid artery (ICA), without the separation of the pterygopalatine artery. The proximal part of CCA and ECA were ligated respectively, after which the distal end of CCA was closed temporarily by the micro artery nip. A small incision was made at the distal end of CCA using ophthalmic scissors at a 45° angle. The sutures were inserted into the CCA through the incision. The thread on the CCA was tied in order to prevent bleeding. After removal of the micro artery nip, the ophthalmic forceps were used in a gradual manner to push the suture. When the end of the suture had entered the CCA branching, the radian was adjusted at the lower right direction and stopped at resistance. After the insertion depth from CCA branching was roughly 16–18 mm (according to animal weight), occlusion of blood vessels was made through the initial terminal of middle cerebral artery to the proximal end in brain, and suture fixed by the thread. The skin was then sewn, with the exposed part of the end of the suture marked. After the ischemia lasted 2 h, the suture was pulled out about 1 cm to allow the ligated end to return to the CCA, which facilitated reperfusion. In the control group, the nylon line was inserted to the rat about 10 mm, with the remaining steps performed as per the model group procedures. During the period of ischemia and 1 h after reperfusion, the body temperature of rat model was maintained at 37 °C ± 0.5 °C. The respiratory secretion was removed in a prompt manner in order to maintain a patent airway. The rats were assigned into 5 groups: control group, WT-MCAO group, miR-195 mimic MCAO group, miR-195^−/−^ MCAO group, and KLF5^−/−^ MCAO group. In the miR-195 mimic MCAO group, miR-195 mimic segments were cloned to vector rAAV2/EGFP and then injected into successful MCAO rat models via tail intravenous injection in accordance with the instructions of the rAAV2/EGFP kit (AAV-006, Beijing Fiveplus Molecular Medicine Institute, Beijing, China). All animal studies were conducted in strict accordance with the recommendation provided by the Guide for the Care and Use of Laboratory Animals of the National Institutes of Health.

### Neurological function score

At the 24th hour after the operation, neurological deficits in the rats were assessed based on the following scoring system as previously reported by Zea Longa: no neurological deficit = 0; failure to fully extend left forepaw = 1; circling to the other side = 2; spontaneous falling to the opposite side when walking = 3; unable to walk spontaneously and became unconsciousness = 4. The higher score obtained; the more serious the animal behavior disorder. The criterion of successful model establishment was that after wakefulness following anesthesia, rat models stood unstably, and turned to one side when carrying the tails, with their left limbs paralyzed. The rat models with 0 point were excluded from the study.

### Triphenyltetrazolium chloride (TTC) staining

The reaction between TTC and succinate dehydrogenase in the normal tissues turned red, whereas it turned pale with succinate dehydrogenase in the ischemic tissues due to the decrease in dehydrogenase activity. The procedures of TTC staining were conducted in accordance with a previously reported method (Xing et al., 2016, Yang et al., 2018). After 3 d, the brain tissues were collected following a neurobehavioral evaluation, then frozen at − 20 °C for approximately 20 min, and subsequently cut into 1.5-mm coronal sections with a sharp blade. The sections were then incubated in 0.5% TTC + Phosphate Buffered Saline (PBS) for 20 min at 37 °C under conditions void of light. After even staining, the sections were placed on the glass plate based on the brain anatomical order and scanned. After the scanned pictures were optimized and processed, the infarct size was analyzed using Image-pro plus software.

### Nissl staining

Whole rat brains were removed and fixed with 4% paraformaldehyde overnight followed by dehydration with sucrose. The dehydrated rat brain was then placed on the sheet iron which was pre-cooled by dry ice. After removal of the excess part of the brain, it was vertically placed on a base which was frozen by optimal cutting temperature (OCT) compound. Next, the brain was embedded, frozen by OCT compound, and cut into sections at 20 μm with the surface then mounted. The procedure of the Nissl staining in hippocampus of the brain was performed in accordance with a previously outlined method (Wang et al., 2017, Peng et al., 2019). After drying for 30 min, the sections were treated with pure water for 10 s and then transferred into cresyl violet acetate for 1–1.5 h under dark conditions. The floating color in the sections was washed off using pure water and subsequently placed in 70, 80 and 95% alcohol for color separation (each for a few seconds). The absence of color fading was considered to represent superiority. The sections were then added into a special color separation solution (1: 1: 1; absolute ethanol, chloroform, ether) for a few seconds. Next, the sections were immersed twice with 100% ethanol (5 min each time), then infused twice with xylene (5 min each time), mounted with a transparent gum, and observed under a fluorescence microscopy. The neurons in the left and right hippocampus of the brain sections of each rat were counted and averaged, with the average value of each group recorded. Each group provided a single value (number of neuronal cells in the length of 200 mm) (Ai et al., 2019).

### Ultrastructure observation by electron microscope

Fourteen days after operation, the rat model was injected intraperitoneally with 1% pentobarbital sodium for anesthesia, followed by chest opening and heart exposure. The left ventricular aorta was rapidly perfused with 200 mL saline and then fixed with 0.1 mol/L PBS containing 2% paraformaldehyde and 2.5% glutaraldehyde for 30 min. The head was promptly cut and the brain tissue sections (containing sensorimotor cortex) 2 mm before and after the optic chiasm were collected. The residual sensorimotor cortex around ischemic foci was separated on an ice table. After preparation of the cerebral cortex sections (1 mm × 1 mm × 1 mm), they were immediately fixed by 3% glutaraldehyde (prepared by 0.1 M PBS) for 3–4 h, washed 3 times with 0.1 mol/L PBS (15 min each time) and fixed with 1% osmium tetroxide for 1 h at 4 °C. The sections were then washed 3 times with 0.1 mol/L PBS (15 min each time), dehydrated with gradient acetone and embedded with Epon812. After optical positioning of semi-thin sections, ultrathin sections (60 nm) were made by Leica ultramicrotome. The sections were subsequently transferred onto a 300-mesh copper screen, and stained by uranyl acetate and lead citrate. The sections were observed, and photographed, with the images analyzed by a Hitachi H-600IV transmission electron microscope (HITACHI, Tokyo, Japan). Quantitative analysis of the Gray type I synaptic interface curvature, number of synapses and postsynaptic density (PSD) was calculated by Image-Pro Plus6.0 software. The Gray type I synapse was characterized by a thick, dense and large postsynaptic membrane with unstructured compact zone in the synaptic gap. The synaptic interface curvature was reflected by the curvature of the joint interface of the synapse. The calculation formula was as follows: curvature = arc length/chord length. The thickness of PSD was measured using the Güldner method (Jones, 1993, Guldner and Ingham, 1980).

### Immunohistochemistry

The rat model was injected with 1% pentobarbital sodium into the abdominal cavity for anesthesia with the brain tissues fixed with 4% paraformaldehyde. The brain tissue sections (containing sensorimotor cortex) 2 mm before and after the optic chiasm were collected and subsequently fixed with 4% paraformaldehyde at 4 °C overnight. The sections were dehydrated by 30% sucrose until they had sunk to the bottom. After quick freezing, the serial coronal sections (30 μm) were constructed. The sections were collected in 0.02 mol/L PBS. Following being heated in an oven at 60 °C for 1 h, the sections were then dewaxed by xylene (YB-5485, Shanghai Yubo Biological Technology CO., Ltd., Shanghai, China) and dehydrated by gradient alcohol. The sections were then soaked in 3% H_2_O_2_ for 20 min in order to eliminate the endogenous peroxidase activity. After being rinsed with PBS, the sections received two antigen repairs, and were then sealed with 10% goat serum for 15 min, incubated with primary antibodies, rabbit anti-rat growth associated protein-43 (GAP-43) (1: 200, ab216497); synaptophysin (SYP) (1: 500, ab53166) and KLF5 (1: 500, ab24331) at 4 °C overnight. The sections were washed 3 times with PBS and incubated with the secondary antibody, biotin-labeled goat anti-rabbit immunoglobulin G (IgG) (1: 1000, ab6721) at 37 °C for 40 min. All the aforementioned antibodies applied were obtained from Abcam, (Cambridge, UK). The sections were then re-washed with PBS, stained for 10 min with diaminobenzidine (DAB, DA1010, Beijing Solarbio Science & Technology Co. Ltd., Beijing, China) and restrained with hematoxylin (H8070, Beijing Solarbio Science & Technology Co. Ltd., Beijing, China). After washing under running water, the sections were subsequently dehydrated, cleared, and mounted with PBS as the negative control (NC). The integral optical density (IOD) values were considered to be indicative of the area and intensity of GAP-43 and SYP immunoreactive products. Three visual fields (200 ×) were randomly selected and photographed around the infarct area in each section. The OD of infarct area was measured by Image-Pr0 Plus 6.0 pathological image analysis system. Three sections were measured from each specimen, and the mean value was recorded.

### Laser capture microdissection (LCM)

A laser capture microscope equipped with laser pressure ejection (PALM Microbeam, Zeiss, UK) was applied to isolate a plurality of individual neuronal cells from the prepared sections (Martuscello et al., 2019, Davis et al., 2019, Thompson et al., 2019). All the manipulations used to capture cells were performed manually on a microscope. The cells were captured and separated according to their respective neuronal size, location and morphology. The cells were automatically cut and separated using 40 × objective lens and cutting control software. After isolation, RNA extraction, amplification and RT-qPCR were performed.

### Flurometric immunosorbent enzyme assay (FIENA)

FIENA was employed for the experiment in accordance with the provided instructions. The cultured cells were rinsed with cold PBS, and then collected after centrifugation. Each sample was lysed with 200 μL lysis buffer in an ice-bath for 1 min, with 100 μL supernatant removed for evaluation. The cells were then added with 100 μL Caspase-3 antibody coating buffer, covered with special adsorption slice at 37 °C for 1 h followed by removal of the coating buffer. Next, the slice was incubated with 200 μL sealing solution for 30 min at room temperature. After the removal of the sealing solution, the slice was washed 3 times with incubated buffer (each for 1 min). The slice was then covered with 100 μL samples at 37 °C for 2 h after which the samples were removed. The slice was subsequently washed with incubated buffer 3 times (each for 1 min). The slice was then covered with substrate reaction solution at 37 °C for 2 h. Time-resolved fluoroimmunoassay instrument was applied to excite the wavelength at 355 nm and release the wavelength at 460 nm. Caspase-3 activity (μm) was calculated based on the instructions provided by the kit.

### TdT-mediated dUTP Nick-end labeling (TUNEL) staining

The brain tissues were made into 5 μm paraffin sections, dewaxed by xylene, hydrated by gradient ethanol. H_2_O_2_ (0.3%) and methanol solution was added to the sections to block endogenous peroxidase at room temperature for 30 min. The sections were then rinsed twice with tris-buffered saline (TBS; each for 5 min). The water around the tissues was removed using filter paper. The sections were then added with the protease K working fluid for 30 min at 37 °C. When cooling down to the room temperature, sections were flushed with twice with TBS for 5 min each and immersed in 0.1% Triton X-100 and sodium citrate solution at room temperature for 5 min. Double distilled water was used to wash the sections twice each for 5 min with the excessive water then dried using filter paper. Next, the sections were stained with TUNEL reaction buffer at 37 °C for 90 min. After cooling down to room temperature, the sections were washed twice with TBS (each for 5 min) with excessive water being removed by filter paper, blocked at 37 °C in normal goat serum for 30 min. After serum removal, the sections were added with peroxidase transforming agent, incubated for 30 min at 37 °C. Then 0.3% H_2_O_2_ and 0.05% diaminobenzidine (DAB) solution was applied to the sections. After the positive nuclei were stained brown, the sections were rinsed with double distilled water in order to terminate the reaction.

### Preparation of oxygen glucose deprivation (OGD) model and virus infection

The rat cerebral cortex cells RCCNC (CBR130669, Celltech Co., Ltd., Shanghai, China) were cultured in an incubator (5% CO_2_, 95% O_2_) with saturated humidity at 37 °C for 6 d. The cells were then grouped into the control (RCCNC cells without virus vector infection and OGD treatment), blank (OGD-treated RCCNC cells without virus vector infection), NC (OGD-treated RCCNC cells with infection of empty virus vector), miR-195 mimic (OGD-treated RCCNC cells with infection of virus vector carrying miR-195 mimic), miR-195 inhibitor (OGD-treated RCCNC cells with infection of virus vector carrying miR-195 inhibitor), small interfering (si)-KLF5 (OGD-treated RCCNC cells with infection of virus vector expressing siRNA against KLF5), and miR-195 inhibitor + si-KLF5 (OGD-treated RCCNC cells with infection of virus vector carrying miR-195 inhibitor and si-KLF5) groups. After 72 h of immersion in medium, the medium was renewed. After the OGD cell ischemic model was developed, the culture medium was renewed with glucose-free Dulbecco’s modified eagle’s medium (DMEM). The plate was then incubated in a low-oxygen incubator (containing 5% CO_2_, 1% O_2_ as well as 94% N_2_) for 1 h at 37 °C for OGD (except the control group). Next, the glucose-free DMEM was replaced with medium (in the presence of glucose). The plate was then cultured in an incubator (containing 5% CO_2_ and 95% O_2_) with saturated humidity at 37 °C for 24 h (reoxygenation).

### Dual luciferase reporter gene assay

MicroRNA.org was employed to predict the target gene of miR-195. Dual luciferase reporter gene assay was performed to validate whether KLF5 was a direct target of miR-195. Based on the sequence of the 3’untranslated region (UTR) of KLF5 mRNA and miR-195, we designed the target sequence and mutant sequence. The target sequence was synthesized with the ends added with endonuclease sites of Xho *I* and Not *I*. The synthetic fragments were cloned into the vector PUC57. After identification of the positive clones, the recombinant plasmid was determined by DNA sequencing, sub-cloned into psiCHECK-2 vector, and then transferred into *Escherichia coli* DH5α cells. After amplification, the plasmids were extracted based on the instructions of the Omega plasmid mini kit (Omega Bio-Tek, Norcross, GA, USA). The cells were then seeded into a 6-well plate at a density of 2 × 10^5^ cells per well and transfected following cell adherence to the wells. After culturing for 48 h, the cells were harvested for subsequent experiments. Luciferase activity of KLF5 3′-UTR altered by miR-195 were measured in accordance with the instructions of the luciferase assay kit (Genecopoeia Inc., Rockville, MD, USA). Fluorescence was assessed by the Glomax 20/20 luminometer (Promega, Madison, WI, USA). All experiments were repeated three times.

### Reverse transcription-quantitative polymerase chain reaction (RT-qPCR)

The total RNA collected from the cells and tissues was isolated using the Trizol one-step method (15,596,026, Invitrogen Inc., Carlsbad, CA, USA) with miRNA isolated using the mirVanaTM miRNA kit (AM1552, Ambion, Austin, TX, USA). An ultraviolet spectrophotometer (DU640, Beckman Coulter, Inc., Chaska, MN, USA) was then employed to evaluate the RNA concentration and purity, with the ratio of A260 to A280 between 1.8 and 2 considered to be indicative of high purity. The RNA (20 μL) was then reversely transcribed into cDNA with the application of the PrimeScript RT reagent Kit (RR047A, Takara Holdings Inc., Kyoto, Japan). RT-qPCR was conducted an ABI 7500 instrument (Applied Biosystems, Foster City, CA, USA) with a SYBR Premix EX Taq Kit (RR420A, Takara Holdings Inc., Kyoto, Japan). Each well was set with 3 duplicate wells. The primers of miR-195, KLF5, and glyceraldehyde-3-phosphate dehydrogenase (GAPDH) were synthesized by Shanghai Genechem Co., Ltd. (Shanghai, China) (Table 1). The Ct value in each well was recorded. U6 was regarded as the internal reference for miR-195, while the internal reference for other genes was GAPDH. The fold changes were calculated using relative quantification (2^-△△Ct^ method).

**Table 1:** Primer sequences used for reverse transcription quantitative polymerase chain reaction

Genes	Sequences
miR-195	Forward: 5′-ATGACAGAAAATGGCCTTCCAGCCT-3’
	Reverse: 5′-TCAGTCCTCAAAGACTTCCAAGAA-3’
KLF5	Forward: 5′-AGCCACCAGAGCGAATCC-3’
	Reverse: 5′-GCCAGCCTATGAGACATTAAGG-3’
GAPDH	Forward: 5′-GCCTTCTCCATGGTGGTGAA-3’
	Reverse: 5′-GGTCGGTGTGAACGGATTTG-3’
U6	Forward: 5′-CTCGCTTCGGCACGCACA-3’
	Reverse: 5′-AACGCTTCACGAATTTGCGT-3’

Note: *miR-195* microRNA-195, *KLF5* Krüppel-like factor 5, *GAPDH* glyceraldehyde-3-phosphate dehydrogenase

### Western blot analysis

Radioimmunoprecipitation assay (RIPA) lysis buffer containing phenylmethyl sulfonylfluoride (PMSF) (R0010, Beijing Solarbio Science & Technology Co. Ltd., Beijing, China) was employed to extract total protein from cells and tissues on ice for 30 min. The protein was centrifuged at 4 °C at 12000 r/min for 10 min to collect the supernatant. The total protein concentration was examined using a bicinchoninic acid (BCA) protein assay kit (23,225, Pierce, WI, USA) and adjusted by deionized water. A total of 50 μg of protein samples were separated by 10% sodium dodecyl sulfate polyacrylamide gel electrophoresis (SDS-PAGE; P0012A, Beyotime Institute of Biotechnolog Shanghai, China) for 2 h at 80 V and transferred onto polyvinylidene fluoride (PVDF) membranes (ISEQ00010, Millipore, Billerica, MA, USA) for 2 h at 110 V. The membranes were blocked with Tris-buffered saline + Tween 20 (TBST) supplemented with 5% skimmed milk for 2 h. The membranes were then incubated with diluted rabbit anti-rat polyclonal antibodies to KLF5 (1: 500, ab24331), JNK (1: 500, ab179461), p-JNK (1: 2000, ab124956), Bcl-2 (1: 500, ab59348), and Bax (1: 500, ab53154) overnight at 4 °C. The membranes were subsequently probed with a horseradish peroxidase-conjugated goat anti-rabbit IgG secondary antibody (1: 2000, ab6721) at room temperature for 1 h, and washed 3 times with PB-Tween 20 (PBST; each for 10 min). The aforementioned antibodies were purchased from Abcam (Cambridge, UK). The membranes were developed under conditions void of light via immersion in the enhanced chemiluminescence (ECL) reagent (WBKLS0100, Millipore, MA, USA), exposed and imaged. The relative protein expression was reflected by the gray value of the target protein band to that of the GAPDH protein band.

### Statistical analysis

All analyses were conducted using SPSS 21.0 software (IBM Corp. Armonk, NY, USA). Data are expressed as the mean ± standard deviation. All experiments were repeated 3 times. The *t*-tests were conducted to determine the statistical significance between two groups while one-way analysis of variance (ANOVA) was performed for comparison among multiple groups. *p* < 0.05 was considered to be indicative of statistical significance.

## Results

### The MCAO rat model is successfully developed

No neurological deficits were detected in the control group, while the rats in the WT-MCAO, miR-195^−/−^ MCAO, miR-195 mimic MCAO and KLF5^−/−^ MCAO groups recovered from anesthesia and exhibited neurological deficits of varying degrees. The scores in the WT-MCAO and miR-195^−/−^ MCAO groups increased significantly (both *p* < 0.05), while the scores in the miR-195 mimic MCAO and KLF5^−/−^ MCAO groups diminished significantly (both *p* < 0.05). The results obtained revealed that the nerve function was obviously damaged after cerebral infarction in rats, and the MCAO model was successfully constructed (Fig. 1).

**Fig. 1:** MCAO rat model was successfully established. ^*^p < 0.05 compared with the control group; *p* < 0.05 compared with the WT-MCAO group; WT, wild type; MCAO, middle cerebral artery occlusion

### Overexpression of miR-195 or loss of KLF5 inhibits cerebral infarction and loss of neuronal cells

TTC staining was applied to determine the infarct volume, in which the infarcted brain tissue was pale, and the normal brain tissue was red. The brain tissue of the control group was red with no signs of pale infarction identified. In comparison with the control group, the brain tissue in the WT-MCAO, miR-195^−/−^ MCAO, miR-195 mimic MCAO and KLF5^−/−^ MCAO groups exhibited different degrees of paling, and also exhibited obvious infarction, and increased infarct volume (all *p* < 0.05; Fig. 2a). Relative to the WT-MCAO group, the infarct volume was increased in the miR-195^−/−^ MCAO group and reduced in the miR-195 mimic MCAO and KLF5^−/−^ MCAO groups (all *p* < 0.05; Fig. 2b). Next, the neuronal cells from the ischemic core and the ischemic boundary zone were separated by LCM to determine the expression of miR-195. The results showed that the expression of miR-195 was significantly increased in the isolated neuronal cells from ischemic boundary zone compared with that from ischemic core zone (all *p* < 0.05; Fig. 2c).

**Fig. 2:** Cerebral infarction size was suppressed in response to overexpression of miR-195 or poor expression of KLF5. **a** TTC staining results of cerebral infarction size in rats of each group; **b** Cerebral infarction size in rats of each group shown by histogram. **c** The expression of miR-195 in the neuronal cells from the ischemic core and the ischemic boundary zone detected by RT-qPCR. ^*^, *p* < 0.05, compared with the control group or the ischemic core zone group; ^#^, *p* < 0.05, compared with the WT-MCAO group; MCAO, middle cerebral artery occlusion; miR-195, microRNA-195; WT, wild type; KLF5, Kruppel-like factor 5; TTC: Triphenyltetrazolium chloride

The results (Fig. 3a, b) of Nissl staining suggested that the neuronal cells in the infarct area and the peri-infarct area were diminished in the ischemic rats of the WT-MCAO, miR-195^−/−^ MCAO, miR-195 mimic MCAO and KLF5^−/−^ MCAO groups when compared to the control group, with the remaining perikaryon shrank, decreased or disappeared neurites, in addition to gradually decomposed or disappeared Nissl bodies. Conversely, the neuronal loss in the miR-195 mimic MCAO and KLF5^−/−^ MCAO groups was significantly decreased, and the neuronal loss in the miR-195^−/−^ MCAO group was increased relative to the WT-MCAO group (all *p* < 0.05). The aforementioned findings showed that upregulated miR-195 or downregulated KLF5 could suppress cerebral infarction and neuronal loss.

**Fig. 3:** Loss of neuronal cells could be suppressed with the overexpression of miR-195 or poor expression of KLF5. **a** Nissle staining results of neuronal cells of rats (400 ×); **b** Number of Nissle stained neuronal cells in rats presented by histogram. ^*^, *p* < 0.05, compared with the control group; ^#^, *p* < 0.05, compared with the WT-MCAO group; MCAO, middle cerebral artery occlusion; miR-195, microRNA-195; WT, wild type; KLF5, Kruppel-like factor 5

### Overexpression of miR-195 or loss of KLF5 promotes synaptic plasticity

An electron microscope was used to observe the ultrastructure of synapse. After 14 d of modeling, the neuronal cells and gliacytes in the control group were identified to be regular in shape, with a large nucleus and complete nuclear membrane structure. The presynaptic and postsynaptic membranes were clearly and completely shaped. The organelles in the presynaptic and postsynaptic areas such as mitochondria and Golgi apparatus exhibited clear and abundant structures with round and uniform synaptic vesicles. The presynaptic terminals gathered a large number of dense and uniform synaptic vesicles. The presynaptic membranes were slightly thickened, and the postsynaptic membranes were evidently thickened. The dense electron-dense materials, long synaptic contact zones, and perforated synapses were all observed. The gliacytes and neuronal cells in the marginal ischemic areas of the ischemic rats from the WT-MCAO, miR-195^−/−^ MCAO, miR-195 mimic MCAO and KLF5^−/−^ MCAO groups were damaged; cells showed edema, and damaged nuclear membrane structures; Heterochromatin increased and accumulated in the nuclei; Synapses disintegrated and decreased with unclear shapes (Fig. 4a, b). The number of synapses, the thickness of PSD and the curvature of synaptic interfaces were remarkably diminished when compared to the control group and they showed an increase in the miR-195 mimic MCAO and KLF5^−/−^ MCAO groups, and a decrease in the miR-195^−/−^ MCAO group in contrast to the WT-MCAO group (all *p* < 0.05; Fig. 4c, d).

**Fig. 4:** Upregulated miR-195 and downregulated KLF5 promoted synaptic plasticity. **a** Electron microscopy images in each group, the red arrow referring to the PSD (10,000 ×); **b** The number of synapses in each group presented by histogram; **c** The curvature of synaptic interfaces in each group presented by histogram; **d** The thickness of PSD in each group as illustrated by histogram; ^*^, *p* < 0.05, compared with the control group; ^#^, *p* < 0.05, compared with the WT-MCAO group; MCAO, middle cerebral artery occlusion; miR-195, microRNA-195; WT, wild type; KLF5, Kruppel-like factor 5; PSD, postsynaptic density

GAP-43 protein was predominately expressed in the cytoplasm and cell membranes were observed to be stained brown. There was no positive staining in the infarction center area, but it was found around the infarction area (Fig. 5a). The positive expression of SYP was primarily located in neuronal cells and neuritis, particularly in the neuritis. The staining was uniform and the neurites were completely arranged in fasciculation (Fig. 5b). The immunohistochemical staining and western blot analysis results indicated that GAP-43 and SYP proteins exhibited higher expression in the miR-195 mimic MCAO and KLF5^−/−^ MCAO groups, and a decline in expression in the miR-195^−/−^ MCAO group when compared to the WT-MCAO group (Fig. 5a-c). The aforementioned results demonstrated that up-regulation of miR-195 promoted GAP-43 and SYP expression, thus enhancing neuronal growth, development, axonal regeneration and synaptic remodeling.

**Fig. 5:** Overexpression of miR-195 enhanced GAP-43 and SYP expression on GAP-43 and SYP expression, thus enhancing neuronal growth, development, axonal regeneration and synaptic remodeling. **a** Immunohistochemical staining results (200 ×) and the OD value presented by histogram of GAP-43 in each group; **b** The immunohistochemical staining results (200 ×) and the OD value presented by histogram of SYP in each group; **c** Western blot analysis of the protein band graph of GAP-43 and SYP and their protein expressions relative to GAPDH presented by histogram; ^*^, *p* < 0.05, compared with the control group; ^#^, *p* < 0.05, compared with the WT-MCAO group; MCAO, middle cerebral artery occlusion; miR-195, microRNA-195; WT, wild type; KLF5, Kruppel-like factor 5; OD, optical density; GAPDH, glyceraldehyde-3-phosphate dehydrogenase; GAP-43, growth associated protein-43; SYP, synaptophysin

### miR-195 negatively regulates KLF5 expression

The online analysis and dual luciferase reporter gene assay were employed to predict and verify the binding correlation between miR-195 and KLF5, the results of which revealed the existence of binding sites between miR-195 and KLF5. Hence, KLF5 was a direct target of miR-195 (Fig. 6a). The luciferase activity of KLF5-Wt in the miR-195 mimic group was reduced in comparison with the NC group (*p* < 0.05, Fig. 6b). Nevertheless, there was no significant difference in relation to the luciferase activity of KLF5-Mut between the NC and miR-195 mimic groups (*p* > 0.05).

**Fig. 6:** miR-195 could negatively regulate KLF5 expression; miR-195 was downregulated while KLF5 was upregulated in ischemic stroke. **a** Predicted binding site of miR-195 on the 3′-UTR of KLF5; **b** Luciferase activity of KLF5-Wt and KLF5-Mut determined by dual luciferase reporter gene assay; **c** Expression of miR-195 and KLF5 in brain tissues in MCAO models; **d** Protein expression of KLF5 in brain tissues in MCAO models; **e** relative expression of miR-195 and KLF5 in RCCNC cells in OGD models measured by RT-qPCR; **f** Protein expression of KLF5 in RCCNC cells in OGD models measured by western blot analysis; **g** Immunohistochemical staining results of KLF5 expression in brain tissues in MCAO models (400 ×); **h** positive rates of KLF5 protein. ^*^, *p* < 0.05, compared with the control group; ^#^, *p* < 0.05, compared with the blank and WT-MCAO groups; MCAO, middle cerebral artery occlusion; miR-195, microRNA-195; WT, wild type; KLF5, Kruppel-like factor 5; NC, negative control; OGD, oxygen glucose deprivation

Next, RT-qPCR and western blot analysis were conducted to measure the expression of miR-195 and KLF5 in MCAO models. The results (Fig. 6c, d) indicated that the mRNA and protein expression of KLF5 elevated and miR-195 expression were downregulated in the WT-MCAO group when compared to the control group (all *p* < 0.05); KLF5 mRNA and protein expression elevated while miR-195 expression exhibited decreases in the miR-195^−/−^ MCAO group, which was opposite when KLF5 mRNA and protein expression declined and miR-195 expression elevated in the miR-195 mimic MCAO group compared with the WT-MCAO group (all *p* < 0.05). The mRNA and protein expression of KLF5 were decreased in the KLF5^−/−^ MCAO group (*p* < 0.05), while the expression of miR-195 exhibited no significant difference in contrast to the WT-MCAO group (*p* > 0.05).

In the OGD models, the RT-qPCR and western blot analysis (Fig. 6e, f) results indicated that the KLF5 mRNA and protein expression raised and miR-195 expression was diminished in the blank group compared to the control group (all *p* < 0.05); The mRNA and protein expression of KLF5 elevated and miR-195 expression reduced in the miR-195 inhibitor group while the mRNA and protein expression of KLF5 decreased and miR-195 expression increased in the miR-195 mimic group relative to the blank group and the NC group (all *p* < 0.05). The si-KLF5 group displayed reduced mRNA and protein expression of KLF5, but no difference was detected regarding the miR-195 expression in contrast to the blank group (*p* > 0.05). In comparison with the miR-195 inhibitor group, miR-195 expression displayed no difference and KLF5 expression reduced in the miR-195 inhibitor + si-KLF5 group (*P* > 0.05). In comparison to the si-KLF5 group, miR-195 expression decreased and KLF5 expression enhanced in the miR-195 inhibitor + si-KLF5 group.

The immunohistochemical staining results of KLF5 (Fig. 6g, h) revealed that the immunoreactivity of KLF5 was predominantly located in the nuclei, and KLF5 expression in the WT-MCAO group was remarkably elevated relative to that of the control group (*p* < 0.05). In comparison to the WT-MCAO group, KLF5 expression was upregulated in the miR-195^−/−^ MCAO group, and downregulated in the KLF5^−/−^ MCAO and miR-195 mimic MCAO groups (all *p* < 0.05). Taken together, miR-195 was lowly expressed while KLF5 was overexpressed in ischemic stroke. miR-195 could negatively regulate KLF5 expression.

### miR-195 inhibits JNK signaling pathway and neuronal apoptosis by downregulating KLF5 expression

The JNK signaling pathway-related protein JNK expression and its phosphorylation were evaluated by western blot analysis. In MCAO models, as depicted in Fig. 7a, b, JNK expression and its phosphorylation were enhanced in the WT-MCAO group versus the control group (*p* < 0.05). In comparison with the WT-MCAO group, the JNK expression and its phosphorylation were potentiated in the miR-195^−/−^ MCAO group and decreased in the KLF5^−/−^ MCAO and miR-195 mimic MCAO groups (all *p* < 0.05;). In OGD models, the JNK expression and its phosphorylation were higher in the blank group and the NC group versus the control group (*p* < 0.05). Relative to the blank group and the NC group, the expression of p-JNK and JNK was diminished in the miR-195 mimic and si-KLF5 groups, while elevated in the miR-195 inhibitor group (all *p* < 0.05). In contrast to the miR-195 inhibitor group, JNK expression and its phosphorylation were reduced in the miR-195 inhibitor + si-KLF5 group (both *p* < 0.05). The JNK expression and its phosphorylation were increased in the miR-195 inhibitor + si-KLF5 group versus the si-KLF5 group (*p* < 0.05; Fig. 7c, d). This highlighted that the overexpression of miR-195 could inhibit JNK signaling pathway by down-regulating KLF5 expression.

**Fig. 7:** miR-195 can inhibit the JNK signaling pathway by down-regulating KLF5 expression. **a** The protein band graph of JNK and phosphorylated JNK in MCAO rats measured by Western blot analysis; **b** Protein expression ratio of JNK/phosphorylated JNK in brain tissues in MCAO rats shown by histogram; **c** The protein band graph of JNK and phosphorylated JNK in RCCNC cells in OGD models measured by western blot analysis; **d** JNK/phosphorylated JNK protein expression ratio in RCCNC cells in OGD models shown by histogram; ^*^, *p* < 0.05, compared with the control group; ^#^, *p* < 0.05, compared with the blank and WT-MCAO groups; MCAO, middle cerebral artery occlusion; miR-195, microRNA-195; WT, wild type; KLF5, Kruppel-like factor 5; NC, negative control; OGD, oxygen glucose deprivation; JNK, Jun N-terminal kinase; p-JNK, phosphorylated-Jun N-terminal kinase; RT-qPCR, reverse transcription-quantitative polymerase chain reaction

Further, western blot analysis was performed to evaluate the expression of apoptosis-related proteins Bax and Bcl-2. In MCAO models, the Bcl-2 expression was diminished, while the Bax expression was elevated in the WT-MCAO group when compared with the control group (*p* < 0.05). Relative to the WT-MCAO group, the Bcl-2 expression was decreased, and Bax expression was enhanced in the miR-195^−/−^ MCAO group while the Bcl-2 expression was increased and the Bax expression was decreased in the KLF5^−/−^ MCAO and miR-195 mimic MCAO groups (all *p* < 0.05; Fig. 8a, b). In the OGD models, the expression of Bcl-2 was diminished, and the Bax expression was increased in the blank group versus the control group (*p* < 0.05). No significant difference was identified between the blank and NC groups (*p* > 0.05). In comparison with the blank group, the Bcl-2 expression was elevated, and the Bax expression was reduced in the miR-195 mimic and si-KLF5 groups while a contrasting trend was observed in the miR-195 inhibitor group (*p* < 0.05). Restored Bcl-2 expression and impaired Bax expression were identified in the miR-195 inhibitor + si-KLF5 group when compared to the miR-195 inhibitor group (*p* < 0.05). Relative to the si-KLF5 group, decreased Bcl-2 expression and increased Bax expression could be observed in the miR-195 inhibitor + si-KLF5 group (*p* < 0.05; Fig. 8c, d).

**Fig. 8:** miR-195 overexpression could decline the expression of KLF5 and inactivate the JNK signaling pathway, thus suppressing neuronal apoptosis. **a** The protein band graph of Bax and Bcl-2 in brain tissues in MCAO rats measured by western blot analysis; **b** Expression of Bax and Bcl-2 protein relative to GAPDH in brain tissues in MCAO rats shown by histogram; **c** The protein band graph of Bax and Bcl-2 in OGD cell models measured by western blot analysis; **d** Expression of Bax and Bcl-2 protein relative to GAPDH in OGD cell models shown by histogram; **e** Results of Caspase-3 activity detection; **f** TUNEL stained cells (400 ×); **g** TUNEL positive cells shown by histogram. ^*^, *p* < 0.05, compared with the control group; ^#,^*p* < 0.05, compared with the blank and WT-MCAO groups; MCAO, middle cerebral artery occlusion; miR-195, microRNA-195; WT, wild type; KLF5, Kruppel-like factor 5; NC, negative control; OGD, oxygen glucose deprivation; Bax, BCL2-associated X protein; Bcl-2, B cell lymphoma-2; TUNEL, TdT-mediated dUTP Nick-End Labeling

The results of Caspase-3 activity detection are depicted in Fig. 8e. In the OGD models, the Caspase-3 activity was elevated in the blank group versus the control group (*p* < 0.05), while no significant difference was detected in the Caspase-3 activity between the blank and NC groups (*p* > 0.05). Caspase-3 activity was diminished in the si-KLF5 group and the miR-195 mimic group, while increased in the miR-195 inhibitor group relative to the blank and NC groups, (all *p* < 0.05). In the OGD models, Caspase-3 activity was reduced in the miR-195 inhibitor + si-KLF5 group when compared to the miR-195 inhibitor alone (*p* < 0.05). In comparison with the si-KLF5 group, Caspase-3 activity was elevated in the miR-195 inhibitor + si-KLF5 group (*p* < 0.05).

TUNEL staining (Fig. 8f, g) was performed for cell apoptosis evaluation. The results indicated that cell apoptosis was potentiated in the WT-MCAO group when compared to the control group (*p* < 0.05). Decreased apoptotic cells were observed in the KLF5^−/−^ MCAO and miR-195 mimic MCAO groups, however, increased apoptotic cells were detected in the miR-195^−/−^ MCAO group relative to the WT-MCAO group (all *p* < 0.05). These data suggested that miR-195 overexpression could downregulate the expression of KLF5 and inhibit the activation of the JNK signaling pathway, thus repressing neuronal apoptosis.

## Discussion

Around the world, approximately 15 million people suffer from stroke ever year, with about 5 million deaths, while another 5 million may be left with life-long disabilities (Rink and Khanna 2011). Thus, the finer molecular mechanisms by which stroke occurs require further elucidation. Accumulating evidence has implicated miRs in the processes of apoptosis, angiogenesis and inflammation in various ischemic diseases (Baczynska et al. 2013). Emerging evidence has demonstrated that miR-195 prevents cerebral ischemic diseases by regulating a variety of key elements (Yang et al., 2018, Cheng et al., 2019). In the current study, we mainly explored the function of miR-195 in ischemic stroke and identified that restoration of miR-195 could induce neuroprotection against ischemic stroke in rat models by suppressing the expression of KLF5 via the JNK signaling pathway.

miR-195 was frequently expressed in the brain and participated in numerous pro-apoptotic and anti-apoptotic processes in cancer cells (Zhou et al. 2013). The upregulation of miR-195 may avoid dendritic degeneration and neuronal death induced by chronic brain hypoperfusion via involvement of the N-APP/DR6/caspase pathway (Chen et al. 2017), and miR-195 was strongly correlated with glioblastoma multiforme, which was known as a very common malignant brain tumor (Lakomy et al. 2011). Moreover, miR-195 can serve as a latent indicator for acute myocardial infarction (Long et al. 2012). It has been well documented that neuronal apoptosis plays a very crucial part in stroke pathophysiology (Liu et al. 2015). Our results illustrated that the overexpression of miR-195 protected nerve function and reduce neuronal apoptosis in MCAO rats with ischemic stroke.

A key observation of our study elucidated that miR-195 could downregulate the expression of KLF5 through repressing the JNK signaling pathway. Through bioinformatics website and the dual-luciferase reporter gene assay, we demonstrated that there was a converse relationship between miR-195 and KLF5. As expected, we identified that suppression of KLF5 expression contributed to neuronal growth and brain plasticity in RCCNC cells induced by OGD and MCAO rats. As a basic transcriptional factor, KLF5 is capable of mediating various physiological and pathological processes involving cell proliferation, apoptosis, migration, differentiation, as well as stemness (Dong and Chen 2009, Ci et al. 2015). Existing literature has highlighted the link between KLF5 inhibition and the cellular transcriptome changes in energy metabolism and neuronal plasticity in the retrosplenial cortex (Poirier et al. 2008). The knockout of other KLF family members, including KLF4 and KLF9, have been shown to help facilitate neurite growth and axon regeneration in retinal ganglion cells following optic nerve injury (Moore et al. 2009). A previous study demonstrated in a damaged nervous system that c-Jun was increased and served as a regulator of transcriptional control in brain function (Raivich 2008). Gennadij Raivich et al. have previously highlighted the inhibitory role of the JNK signaling in neurite outgrowth (Raivich and Makwana 2007). Lorena Soares et al. also concluded that depression of the JNK signaling potentiates regrowth in the injury site and also boosts axonal regeneration (Soares et al. 2014). A previously conducted study demonstrated that JNK blocking protects oxygen species from increasing and mitochondrial dysfunction, thus may serve as a promising therapeutic target of I/R-induced cardiomyocyte death (Chambers et al. 2013). Inhibition of the JNK signaling pathway has been reported to be a beneficial factor in the prevention of neuropathic pain, ultimately playing a promotive role on axon sprouting after peripheral nerve injury (Manassero et al. 2012). KLF5 has been shown to accelerate cell apoptosis and decrease esophageal squamous cell survival by activating the JNK signaling pathway (Tarapore et al. 2013). A corroborating study revealed that the interactions of KLFs and kinases in the MAPK family were linked to the axon growth and regeneration (Apara and Goldberg 2014). Baczynska. Akintomide Apara et al. highlighted the cooperation between KLF9 and JNK3 caused failure on axon growth and regeneration (Apara et al. 2017).

Moreover, our results demonstrated that miR-195 could up-regulate GAP-43, SYP, and Bcl-2 expression, down-regulate Bax expression via the JNK signaling pathway, thereby promoting neuronal growth, development, axonal regeneration and synaptic remodeling. Activation of JNK was shown to aid in elevating the expression of Bax and decreasing the expression of Bcl-2, thereby inducing neuronal cell apoptosis (Lu et al. 2014). Tumor necrosis factor-α could inhibit axonal transport of mitochondria and SYP by stimulation of JNK (Stagi et al. 2006). GAP-43, a neuronal phosphoprotein, plays an essential role in the development of axonal outgrowth from the beginning to the remodeling of neural contacts (Takahashi et al. 2006). In the current study, we identified that GAP-43 was up-regulated after ischemic stroke owing to the stress response of brain for neuro-protection. Consistent with our results, a previous study has revealed that following brachial plexus injury, GAP-43 was elevated in anterior horn motoneurons of the spinal cord (Chen et al. 2010).

## Conclusions

Taken together, the key findings of our study highlighted miR-195 as an important mediator of neuronal apoptosis induced by cerebral ischemia. Hence, treatment strategies targeting miR-195 could be performed to suppress neuronal apoptosis and enhance brain plasticity by inhibiting KLF5 and JNK signaling pathway after ischemic stroke in rat models (Fig. 9). We speculate that it may be possible to recruit miR-195 as a novel ischemic stroke target for precision therapy on the foundation of the function and mechanism of miR-195 clarified in this study. Additional investigations are necessary in order to identify other potential targets of miR-195 and its functions in the modulation of ischemic stroke biology.

**Fig. 9:** The mechanism investigation of miR-195 in different stroke mediators, with a particular emphasis on the KLF5/ JNK axis. Our findings suggested that treatment strategies targeting miR-195 could be performed to suppress neuronal apoptosis and enhance brain plasticity by inhibiting KLF5 and JNK signaling pathway after ischemic stroke in rat models

## Data Availability

The datasets generated/analyzed during the current study are available.

## Abbreviations

ANOVA: Analysis of variance
BCA: Bicinchoninic acid
CA: Carotid artery
CCA: Right CA
DMEM: Dulbecco’s modified eagle’s medium
FIENA: Flurometric immunosorbent enzyme assay
ICA: Internal carotid artery
IOD: Integral optical density
JNKs: c-Jun N-terminal kinases
MCAO: Middle cerebral artery occlusion
MCAO: Middle cerebral artery occlusion
MiRs: microRNAs
NC: Negative control
OGD: Oxygen deprivation
OGD: Oxygen glucose deprivation
PBS: Phosphate buffered saline
PVDF: Polyvinylidene fluoride
RIPA: Radioimmunoprecipitation assay
SD: Sprague Dawley
TTC: Triphenyltetrazolium chloride
TUNEL: TdT-mediated dUTP nick-end labeling
